The article "Automated Detection Model Based on Deep Learning for Knee Joint Motion Injury due to Martial Arts" was published in 2022. Journal: Comput Math Methods Med.

# Automated Detection Model Based on Deep Learning for Knee Joint Motion Injury due to Martial Arts

**DOI:** 10.1155/2022/3647152

**Published:** 2022-05-17

**Authors:** Meng Xue, Yan Liu, XiaoMei Cai

**Affiliations:** ^1^Jiangmen Polytechnic, GuangDong, 529000, China; ^2^Department of Orthopedic Surgery, Jiangmen TCM Affiliated Hospital of Jinan University, GuangDong, 529000, China; ^3^JiangMen Chinese Medical College, GuangDong, 529000, China

## Abstract

**Objective:**

Develop a set of knee joint martial arts injury monitoring models based on deep learning, train and evaluate the model's effectiveness.

**Methods:**

This paper mainly collects knee MRI images of 1546 patients with knee joint martial arts injuries from 2015 to 2020. Through manual annotation, the data set is divided into six categories: meniscus injury, tendon injury, ligament injury, epiphyseal cartilage injury and synovial joint capsule loss. The human knee collaborative MRI image database is established, and the data set is divided into the training and validation sets. And test set. Establish a deep neural network, train the model using the training set and validation set, locate the knee joint injury location, and classify the specific injury type. The model's validity was validated using the test set, and the model's sensitivity, specificity, and mean accuracy for detecting lesions were evaluated.

**Results:**

In the test set, the accuracy of meniscus injury, tendon injury, ligament injury, bone and bone cartilage injury and synovial joint capsule injury were 83.2%, 89.0%, 88.0%, 85.9%, 85.6% and 83.5%, respectively, and the overall average accuracy value was 86.0%. The sensitivity and specificity of the model were 91.3% and 87.3%, respectively.

**Conclusion:**

The application of the deep learning method in the classification and detection of knee joint martial arts injuries can significantly improve the diagnosis effect, reduce the diagnosis time and misdiagnosis rate, and provide decision support for surgery.

## 1. Introduction

In the teaching and training of martial arts, to achieve fast reaction speed and movement speed, athletes have high requirements on the explosive power of lower limbs; athletes need to complete quick knee bend, knee extension, half knee bend and other movements, which cause a lot of local load on the knee joint, easy to lead to a common knee injury. According to statistics, the prevalence of knee osteoarthritis in Chinese wushu athletes is as high as 15.6% [1].

Medically, knee lesions are usually diagnosed by magnetic resonance imaging (MRI). MRI can clearly show articular cartilage and bone areas and is typically segmented layer by layer by an experienced physician [2]. However, due to the relatively complex anatomical structure of the knee joint, and the injury often involves multiple tissue parts, the diagnosis is challenging, and the phenomenon of missed diagnosis usually occurs.

In recent years, with the development and application of convolutional neural networks in medical image analysis, deep learning-based diagnosis has become a feasible method in medical image segmentation [3].

With the development and application of convolutional neural networks in medical image analysis, deep learning-based diagnosis has become a feasible method in medical image segmentation.

In terms of knee imaging application, four types of parts were to be divided: femur bone (FB), femur cartilage (FC), Tibia bone (TB) and Tibia cartilage (TC) [4]. Due to the differences in shape and size of different parts, it is difficult for conventional image recognition algorithms to identify multiple factors simultaneously. Therefore, few diagnosis methods of knee joint lesions are combined with deep learning methods.

This paper, based on U-net codification and decoding architecture, multi-scale context feature extraction module and multi-output fusion module, is designed for segmentation targets of different sizes in knee MRI. Feature reuse is strengthened [5]. The cascade U-net was proposed for knee joint image segmentation. The knee MRI image library was used to train and verify its effectiveness.

## 2. Methodology

The U-net used in this paper is an advanced feedforward neural network [6]. Feedforward neural network, also known as a multilayer perceptron, is a one-way multilayer artificial neural network. Data information is transmitted to the next layer through the upper layer, and the knowledge of the next layer does not influence or feedback on the upper layer [7].

Due to the complex structure of the knee joint and the structural imbalance of different tissue sizes, this paper adopted a cascaded U-net network framework with expanded functions and flexibility for multi-mode segmentation recognition of human knee MRI.

### 2.1. Basic U-Net Model

U-net is essentially a codec model, as shown in Figure 1.

In the coding stage, the network extracts the feature information of the image through the cascaded convolution module. It reduces the resolution through the maximum pooling operation of the feature graph to increase the receptive field of the convolution operation and obtain more global information [8].

In the decoding stage, the corresponding design replaces the maximum pooling operation with a deconvolution operation to restore the resolution of the feature map. At the same time, the number of channels in each small module is halved.

The core operation in the U-net network is to introduce a jump connection between the encoding and decoding layers to reduce the loss of underlying feature information caused by the pooling operation in the encoding stage. The high-level features are helpful for pixel classification, while the low-level features help generate acceptable boundaries. The jump connection directly splices the low-level detail features and high-level semantic features of corresponding stages in the coding-decoding layer. It then carries out feature compression and fusion through the convolution operation, finally achieving high-quality segmentation.

### 2.2. Cascading U-NET Model

Although U-net has achieved excellent results in biomedical image recognition, there is still room for improvement. Based on the traditional U-net, this paper adds the segmentation network structure, takes the network positioning and pruning of the U-net as the input, and obtains the accurate segmentation result by updating the network training parameters [9]. Therefore, this paper mainly makes the following improvements based on the structure of the positioning network.

#### 2.2.1. Improved down Sampling

In the location network, this paper uses the mode of maximum pooling to construct the pooling layer for down-sampling. This down-sampling mode is conducive to extracting powerful features such as edges. It can strengthen the translation invariability of network features so that high-level features have a larger receptive field [10].

Although the pooling operation may eliminate some unimportant semantic features in feature extraction, it will also delete some significant features. To solve this problem, this paper introduces a convolution layer with a convolution kernel size of 3 × 3 × 3 and a step size of 2. It adds an LReLU activation function layer to replace the original pooling layer. This down-sampling method, which uses convolution operation instead of pooling operation, can reduce the input image's resolution, reduce the input signal's size, and increase the receiving field of the features in the subsequent network layer to expand the receptive field.

Convolution layer under-sampling, besides can realize the primary function of the pooling layer, still can keep the input image for more details, more semantic features are extracted. In addition, using the convolution layer to replace the pooling layer for down-sampling can reduce the amount of convolution computation and reduce the memory occupied by the network in the training process [11].

#### 2.2.2. Residual Module

To avoid gradient dispersion and gradient explosion caused by the too high depth of the network model and to further improve the training efficiency and generalization ability of the model, the residual mechanism is introduced to optimize the model.

The residual mechanism is put forward as the original is to solve the deep web layer caused by the increase in the number of network degradation [12, 13]; introducing a residual block can effectively control the gradient diffusion problems, no more parameters are presented at the same time, due to the residual is compared commonly small, residual learning will be more accessible, further strengthened the network characteristic expression ability, improve the network performance.

Figure 2(a) shows the introductory module in U-net, and Figure 2(b) shows the residual module that combines the Batch Normalization (BN) operation. The activation function used is ReLU. Since the dimension changes occurred in the residual module, that is, the number of channels in the input and the number of channels in the output do not match and cannot be directly added, the number of channels is transformed by 1 × 1 convolution, and at the same time, the convolution of 1 × 1 does not introduce too many parameters [14–16].

#### 2.2.3. Extended Convolution Module

In a U-NET network, maximum pooling is used to conduct a downsampling operation on a feature graph, which can increase the receptive field of convolution operation while maintaining a small convolution kernel and losing spatial location information to a certain extent [17]. Therefore, an extended convolution mechanism is introduced in this paper, as shown in Figure 3.

Figure 3(a) shows a two-dimensional convolution with a kernel size of 3, expansion rate of 1 and step size of 1, which is equivalent to conventional convolution. The receptive field is a 3 × 3 region, and the number of parameters is 9.  Figure 3(b) shows a convolution kernel size of 3 and an expansion rate of 2. For the two-dimensional convolution with a step size of 1, except for the position of the blue dot, the weight of other places is 0. Although the number of parameters is still 9 at this time, the size of its receptive field is 7 × 7.

#### 2.2.4. Deep Supervision Mechanism

In this paper, the segmentation network introduces depth supervision mechanism to the hidden layer in the up sampling expansion path, and carries out depth supervision for the last three layers with different sizes, respectively, and outputs the feature information of the hidden layer to the output layer [18].

This paper uses the deep supervision mechanism, does not need to introduce additional with the objective function, supervision is directly through the layer for convolution operation, get the characteristics of the corresponding category information, will be on the characteristics of the deep category information sampling, and the adjacent shallow overlay, feature category information through step by step a repeated operation, finally get an output feature class is used to calculate the objective function. By establishing in-depth supervision of the hidden layer, the hidden layer features are directly extracted, and the semantic feature information of the hidden layer is effectively retained. Meanwhile, the gradient dispersion problem can be effectively controlled and the network performance can be improved through sufficient training of the shallow layer network. The basic structure of depth supervision mechanism is shown in Figure 4.

### 2.3. Experimental Settings

#### 2.3.1. MRI Classification and Labeling of Knee Joint

According to the clinical diagnostic criteria of MRI of knee joint, knee joint injury was classified into 6 categories and 21 items by location, including all common lesions of sports-related knee joint injury, including:(1) meniscus injury (meniscus I ~ II degree injury, meniscus III degree injury); (2) Tendon injury (quadriceps tendon injury medial femoris tendon injury, lateral femoris tendon injury, gastrocnemius intra or lateral head tendon injury, popliteal tendon injury); (3) ligament injury (anterior cruciate ligament injury, posterior cruciate ligament injury, medial collateral ligament injury, lateral collateral ligament injury, ballad ligament injury, iliotibial band injury); (4) bone and osteochondral damage (osteomalacia, bone marrow edema, exfoliative osteochonitis); (5) synovial capsule injury (joint effusion, synovitis); (6) Peripheral soft tissue injury (subcutaneous fasciitis, lipoedema, popliteal cyst) [19].

In this paper, MRI of patients with martial arts injury of knee joints from 2015 to 2020 was screened. After comparative analysis, repetitive and poor quality data were removed, and 1546 MRIwas finally obtained. For each MRI, the location and type of lesions in the image were located by manual labeling. The annotation results showed that among the 1546 MRI images, there were 1242 cases of meniscus injury, 29 cases of tendon injury, 254 cases of ligament injury, 557 cases of bone and bone cartilage injury, 1494 cases of synovial joint capsule injury, and 340 cases of soft tissue injury. The annotation results are shown in Table 1.

#### 2.3.2. Data Preprocessing

By observing the annotation results, we found that the vast majority of knee joint lesions involved two or more combined injuries. At the same time, among different types of injuries, synovial joint capsule injury accounted for the highest proportion (96.6%), while tendon injury accounted for the lowest proportion (1.9%).

At the same time, to further improve the model's generalization ability, we divide the training set and the test set by cross-validation. First, divide the original data into ten equal pieces, ensuring that each piece has the same proportion of different types of data as the original data. During each training, one sample is selected as the test set and the rest as the training set. Since the data of the training set and the test set do not intersect, the over-fitting phenomenon can be avoided to a certain extent.

#### 2.3.3. Judgment Criteria

The prediction result of the model includes two parts, one is the location of lesion, the other is the prediction of lesion type.

The Intersection-over-Union (IOU) was used as the criterion for locating the lesion. Intersection-over-Union is a concept used in object detection. It is the overlap rate of candidate bound and ground truth bound generated, that is, the ratio of their intersection to union. The calculation formula of cross ratio is shown in Equation (1).

(1) $$\begin{array}{c} IOU=\frac{area\left(C\right)\cap area\left(G\right)}{area\left(C\right)\cup area\left(G\right)} \end{array}$$

In the formula, *area (C)* and *area (G)*, respectively, represent the lesion regions predicted by model and manually labeled. The larger the VALUE of IOU is, the higher the fitting degree of the lesion location predicted by the model and the artificially labeled lesion location is. In this paper, we define that when the IOU value is greater than 0.35, the model's lesion location prediction is successful.

The sensitivity, specificity, F1 and average accuracy values commonly used in the classification algorithm were used to evaluate the model for the prediction of lesion types.

Since the model prediction is divided into two parts, we define that only when the lesion location and lesion type are predicted successfully, the model belongs to the classification success, and calculate relevant statistical data based on this.

In order to compare the model performance, this paper takes the traditional U-net model as the benchmark and uses the same data set and training method to analyze and compare the predicted results.

## 3. Experimental Results

Through training, the effect of lesion recognition of cascaded U-NET model and traditional U-NET model is shown in Figure 5.

In Figure 5, the red, green and yellow boxes, respectively, represent the cascade U-NET model, the traditional U-NET model and the manually identified lesion regions, and Case1 to Case 6, respectively, represent the six lesion types mentioned above.

Through observation, the focus area identified by the cascade U-net model is basically the same as the focus area identified by manual annotation, and the model is more accurate in area size than manual annotation. The traditional U-net model can roughly identify the location of the lesion, but the area is large, and there is a certain gap in accuracy compared with the cascaded U-net model. The performance parameters of the two models are shown in Table 2.

In Table 2, the left side represents the recognition effect of the cascading U-net model, and the right side represents the recognition effect of the traditional U-net model.

Through the analysis of the data in the table, it can be found that in the recognition of different types of lesions, the indicators of the cascade U-NET are slightly higher than the traditional U-NET model. In the aspect of ligament injury, the recognition effects of the two models were basically equal, which may be due to the fact that the sample data of ligament injury were few, and the over-sampling model had a higher recognition intensity for such samples. The experimental results show that the cascaded U-NET model has considerable feasibility in the field of knee joint medical image recognition, and has significantly improved performance compared with the traditional model.

## 4. Discussion

The strenuous exercises and activities of wushu determine that it is more likely to cause sports injuries; according to the investigation, wushu athletes' knee joint injuries are more serious. In other professions, such as athletes, soldiers, etc., common knee injury is also higher due to the accumulation of exercise load.

At present, the diagnosis of knee joint injury mainly relies on manual recognition MRI. Due to the complex structure of the knee joint, different parts to be identified differ significantly in shape and size. Manual identification takes a long time, with low accuracy, and sometimes the phenomenon of missed diagnosis and misdiagnosis occurs.

In recent years, deep learning has developed rapidly and has been widely used in the medical field. Deep learning has been used to segment human organs and reconstruct human structures. In medical imaging, deep learning model can be trained to replace manual recognition of human characteristics and provide a reference for manual diagnosis.

In this paper, the deep learning algorithm is combined with knee MRI, and the improved cascade U-net model is used to identify the site and type of knee lesions. Finally, good results are achieved on the test data set. Compared with the traditional deep learning model and manual labeling method, it has specific clinical application value.

## 5. Conclusion

In this paper, we use deep learning algorithms combined with knee MRI diagnosis. Improvements have been made to the traditional U-NET model to improve training efficiency and model efficiency. Compared with the traditional manual labeling method, there is a certain improvement. In the test data set, the average recognition accuracy of the model reached 86.0%, and it could accurately identify the location of lesions and classify the types of lesions, indicating that the model has high application value in medicine and is worthy of further development and research.

## Figures and Tables

**Figure 1:** Basic U-net frame.

**Figure 2:** U-net based on (a) basic module and (b) residual module.

**Figure 3:** The receptive field of detailed convolution based on (a) 3 × 3 and (b) 7 × 7.

**Figure 4:** Deep supervision structure.

**Figure 5:** Effects of different models on the identification of lesions.

**Table 1:** Statistics table of knee joint image samples.

Injured part	Sample size	Proportion	Label
Meniscus	1242	80.3%	1
Tendon	29	1.9%	2
Ligamentous	254	16.4%	3
Bone and apical cartilage	557	36.0%	4
Synovial capsule	1494	96.6%	5
Soft tissue	340	22.0%	6

**Table 2:** Identification accuracy of different models.

Injured part	Sensitivity	Specificity	F1 value	Mean accuracy
Meniscus	95.5/93.7	61.5/60.1	74.9/73.5	83.2/80.3
Tendon	91.3/91.3	87.3/87.2	89.2/89.1	89.0/89.0
Ligamentous	91.1/89.8	83.5/82.5	87.0/85.6	88.0/85.7
Bone and apical cartilage	88.4/87.5	87.6/86.7	88.0/87.1	85.9/85.0
Synovial capsule	91.2/89.4	74.7/73.5	82.3/80.7	85.6/82.5
Soft tissue	86.1/85.2	85.8/84.8	85.9/84.9	83.5/82.3

## Data Availability

The image data used to support the findings of this study have been deposited in the I Do Imaging (IDI) dataset (https://idoimaging.com/home).
